# An Improved Chicken Swarm Optimization Algorithm for Solving Multimodal Optimization Problems

**DOI:** 10.1155/2022/5359732

**Published:** 2022-11-22

**Authors:** Jianhui Liang, Lifang Wang, Miao Ma

**Affiliations:** ^1^School of Computer Science, Northwestern Polytechnical University, Xi'an 710072, China; ^2^School of Applied Science and Technology, Hainan University, Dan Zhou 571737, China; ^3^School of Computer Science, Shaanxi Normal University, Xi'an 710062, China

## Abstract

To solve the premature convergence problem of the standard chicken swarm optimization (CSO) algorithm in dealing with multimodal optimization problems, an improved chicken swarm optimization (ICSO) algorithm is proposed by referring to the ideas of bacterial foraging algorithm (BFA) and particle swarm optimization (PSO) algorithm. First, in order to improve the depth search ability of the algorithm, considering that the chicks have the weakest optimization ability in the whole chicken swarm, the replication operation of BFA is introduced. In the role update process of the chicken swarm, the chicks are replaced by the same number of chickens with the strongest optimization ability. Then, to maintain the population diversity, the elimination-dispersal operation is introduced to disperse the chicks that have performed the replication operation to any position in the search space according to a certain probability. Finally, the PSO algorithm is integrated to improve the global optimization ability of the algorithm. The experimental results on the CEC2014 benchmark function test suite show that the proposed algorithm has good performance in most test functions, and its optimization accuracy and convergence performance are also better than BFA, artificial fish swarm algorithm (AFSA), genetic algorithm (GA), and PSO algorithm, etc. In addition, the ICSO is also utilized to solve the welded beam design problem, and the experimental results indicate that the proposed algorithm has obvious advantages over other comparison algorithms. Its disadvantage is that it is not suitable for dealing with large-scale optimization problems.

## 1. Introduction

The multimodal optimization problem is a complex function optimization problem with one or more local extrema [1]. In practical applications, there are many multimodal optimization problems, such as parameter estimation and identification of models [2, 3], engineering structure optimization, welded beam design [4], and medical diagnosis [5]. It is difficult to find the global optimum because there are many local extrema in the multimodal optimization problem. Therefore, it is of very importance to study efficient and reasonable algorithms [6, 7].

The swarm intelligence optimization algorithm is a kind of bionic random search algorithm which can solve complex optimization problems by imitating the ecosystem mechanism in nature. Because of its strong global search ability, high efficiency, and insensitivity to initial values, it has been widely concerned by relevant researchers [8–10]. At present, hundreds of algorithms based on swarm intelligence have emerged, such as genetic algorithm (GA) [11], particle swarm optimization (PSO) algorithm [12], bacterial foraging algorithm (BFA) [13], and artificial fish swarm algorithm(AFSA) [14]. In the swarm intelligence optimization algorithm, there are no individuals with centralized control, and the interaction between individuals is extremely simple, but they have the ability to solve complex problems in a short time, which makes them very suitable for solving complex optimization problems in practice. Moreover, the swarm intelligence optimization algorithm does not need the gradient information of the optimization problem, so it belongs to the nongradient optimization algorithm. Therefore, it has a wide range of applications [15, 16]. At present, it has been applied in optimization calculation [17, 18], workshop scheduling [19, 20], image engineering [21], network structure optimization [22], vehicle routing problem [23], control of teleoperating systems, and other fields [24].

As a kind of swarm intelligent algorithm, the chicken swarm optimization (CSO) algorithm was proposed by Meng et al. in 2014 [25]. Due to its good stability and global search ability, the algorithm has attracted extensive attention since it was proposed and has been successfully applied in some fields [26, 27]. Liang et al. combined the CSO algorithm with the pulse-coupled neural network for image segmentation. The experimental results show that this method has obvious advantages in convergence speed and segmentation accuracy [28]. Cristin et al. combined the CSO algorithm with the deep neural network for the classification of brain tumors and achieved good performance in terms of accuracy, specificity, sensitivity, and so on [29].

Although the CSO algorithm has shown good performance in solving many benchmark problems and practical problems, it also has some inherent shortcomings, such as premature convergence and falling into local extrema. Therefore, researchers have proposed many improved algorithms. At present, the improvement of the CSO algorithm can be mainly classified into three categories as follows:

1. *Combination with other swarm intelligent algorithms.* For example, Li et al. improved the search ability of the CSO algorithm by integrating the operation of gray wolf optimization algorithm and PSO algorithm into the CSO algorithm. The experimental results show that the algorithm is superior to other basic swarm intelligent algorithms in accuracy, convergence speed [30], etc. Sampath fine-tuned the solution of the CSO algorithm by introducing the differential evolution algorithm to avoid premature convergence and applied the proposed algorithm to solve routing problems [31].
2. *Modification of position update formulas of the chicken swarm.* For example, Gu et al. improved the CSO algorithm by introducing an adaptive update factor and designing the inertia weight and successfully applied it to parameter estimation of the Richards model [32]. Considering that the imbalance between the diversity and intensification of the population may affect the performance of the CSO algorithm, Lin et al. proposed an improved CSO algorithm by modifying the position update formulas of the roosters and hens. Experiments show that this algorithm has obvious advantages over other swarm intelligent algorithms in terms of optimization accuracy and robustness [33].
3. *Multiobjective CSO algorithm.* In order to solve the configuration problem of electric vehicle charging stations, Deb et al. proposed a new hybrid multiobjective CSO algorithm based on pareto optimization. The effectiveness of the algorithm is verified on some multiobjective benchmark problems and the electric vehicle charging station configuration problem [34].

The performance of the aforementioned swarm intelligence optimization algorithms has been improved to a certain extent, but there are still some disadvantages. For example, the literature [18] introduced the differential evolution strategy and quantum behavior into the bird swarm algorithm. Although the convergence speed of the algorithm was enhanced, the problem of premature convergence still existed. In the literature [30], several improved factors are introduced into the position update formulas of the chicken swarm, which improves the ability of the algorithm to jump out of the local extrema to a certain degree. But the optimization accuracy still needs to be further improved.

To solve the abovementioned problems, in this paper, an improved chicken swarm optimization (ICSO) algorithm is proposed which combines the idea of PSO with the replication and elimination-dispersal operations of BFA. More specifically, our contributions are as follows:

1. The replication operation of BFA is applied to the chicks with the weakest optimization ability to inherit the optimal food source in the whole chicken swarm, which is profitable to enhance the depth search ability of the algorithm.
2. The chicks are dispersed to any position in the search space according to a certain probability by using the elimination-dispersal operation of BFA, which is beneficial to improve the population diversity.
3. The idea of PSO is integrated to improve the global search ability of the algorithm. The experimental results on CEC2014 standard function test suite preliminarily show that this algorithm has obvious advantages over other swarm intelligent algorithms in optimization accuracy and convergence performance [35]. In addition, compared with other comparison algorithms, it also obtains competitive results in solving the welded beam design problem.

## 2. CSO Algorithm

The CSO algorithm is a meta-heuristic optimization algorithm that simulates the foraging behavior of roosters, hens, and chicks in nature. The characteristics of the algorithm are as follows:

1. *Correspondence with the optimization problem*. The algorithm regards several randomly generated positions in the solution space of the optimization problem as several chickens, and the food source of each chicken is measured by the fitness function value of the corresponding optimization problem.
2. *Hierarchical order, that is, the role assignment of the chicken swarm.* The whole chicken swarm is composed of four roles, namely, the roosters, hens, chicks, and mother hens. Their role assignment is based on the content of food sources. The rooster has the best food sources, the hens take the second place, the food sources of the chicks are the worst, and the mother hens are randomly selected from the hens.
3. *Subgroup division.* During the whole foraging process, the chicken swarm is divided into several subgroups. The number of subgroups is determined by the number of the roosters, because each subgroup is composed of a randomly selected rooster, several hens, and chicks, and there is at least one hen in each subgroup.
4. *Relation of dependence.* In the foraging process of the chicken swarm, the chicks follow the chicks' mothers (mother hens) and the hens follow the roosters in their subgroups to forage for food. They can also steal the good food sources found by other subgroups at random.
5. *Information exchange.* The hierarchical order of the chicken swarm and the mother-child relationship between the mother hens and the chicks will be updated after several iterations. The information exchange between subgroups will be realized through continuous role assignment.
6. *Parallel optimization.* The whole chicken swarm can realize parallel optimization through the division of labor and cooperation mechanism between subgroups, quickly find the best food sources, and then obtain the solution to the optimization problem. The formulas used by chickens with different roles in foraging are given below.

The formula used by the roosters in foraging is as follows:

(1) $$\begin{array}{c} X_{i,j}\left(t+1\right)=X_{i,j}\left(t\right)\times \left(1+\text{Randn}\left(0,\sigma^{2}\right)\right)\text{j}\in \left[1,\text{dim}\right], \end{array}$$

(2) $$\begin{array}{c} \sigma^{2}=\left\{\begin{array}{cc} 1 & f_{i}\leq f_{k}\\ \exp\left(\frac{\left(f_{k}-f_{i}\right)}{\left|f_{i}\right|+\varepsilon }\right) & f_{i}>f_{k} \end{array}\right)i,k\in \left[1,rNum\right],k\neq i, \end{array}$$

where *X*_*i*,*j*_(*t*) represents the position of the *i*th rooster in the *t*-th iteration, and dim is the dimension of the optimization problem. Randn(0, *σ*^2^) is a normal distribution with a mean value of 0 and a standard deviation of *σ*^2^. *ε* is a very small number that can be expressed by the computer, which is used to avoid the situation that the denominator is 0 in the formula. *f*_*k*_ represents the content of the food source of any other rooster which is different from the *i*^th^ rooster. *rNum* represents the number of roosters.

The formula used by the hens in foraging is as follows:

(3) $$\begin{array}{c} X_{i,j}\left(t+1\right)=X_{i,j}\left(t\right)+{\text{c}}_{1}\times \text{Rand}\times \left(X_{r_{1},j}\left(t\right)-X_{i,j}\left(t\right)\right)+{\text{c}}_{2}\times \text{Rand}\times \left(X_{r_{2},j}\left(t\right)-X_{i,j}\left(t\right)\right), \end{array}$$

(4) $$\begin{array}{c} c_{1}=\exp\left(\frac{\left(f_{i}-f_{r_{1}}\right)}{\left(abs\left(f_{i}\right)+\varepsilon \right)}\right), \end{array}$$

(5) $$\begin{array}{c} c_{2}=\left(f_{r_{2}}-f_{i}\right), \end{array}$$

where *X*_*i*,*j*_(*t*) is the position of the *i*^th^ hen in the *t*-th iteration. *Rand* is a random number function with a value range of (0, 1). *X*_r1,*j*_(*t*) is the position of the rooster which is in the same subgroup as the *i*^th^ hen. *X*_r2,*j*_(*t*) is any chicken randomly selected from the whole chicken swarm, which is different from the *i*^th^ hen, and *r*_1_ ≠ *r*_2_.

The formula used by the chicks in foraging is as follows:

(6) $$\begin{array}{c} X_{i,j}\left(t+1\right)=X_{i,j}\left(t\right)+FL\times \left(X_{m,j}\left(t\right)-X_{i,j}\left(t\right)\right), \end{array}$$

where *X*_*i*,*j*_(*t*) represents the *i*th chick, and *X*_*m*,*j*_(*t*) is the position of the chick's mother. *FL* ∈ (0, 2) is a following coefficient that the chick follows the chick's mother to search for food.

The corresponding basic flowchart is shown in Figure 1.

## 3. The Proposed Algorithm

Aiming at the premature convergence of the standard CSO algorithm in solving multimodal optimization problems, an ICSO algorithm is proposed in this paper. Considering that the chicks have the weakest optimization ability in the whole chicken swarm, the algorithm improves the foraging behavior of the chicks by referring to the reproduction and elimination-dispersal operations of BFA. At the same time, considering that the PSO algorithm has good global search ability, on the basis of individual division of labor and cooperation optimization mechanism of the CSO algorithm, a hybrid CSO algorithm is constructed to enhance the global search ability of the algorithm by integrating the PSO algorithm.

### 3.1. CSO Algorithm with Reproduction and Elimination-Dispersal Operations (RECSO Algorithm)

In the standard CSO algorithm, chicks are the most vulnerable group. Therefore, in order to improve the depth search ability of the algorithm, this paper introduces the reproduction and elimination-dispersal operations of BFA into the chicks' foraging behavior, and a RECSO algorithm is proposed. Firstly, in the role update process of the chicken swarm, the replication operation of BFA is introduced to replace the chicks with the same number of chickens with the strongest optimization ability. Through this behavior, the depth optimization speed of the chicken swarm can be accelerated. At the same time, in order to maintain the population diversity, the elimination-dispersal operation is introduced to disperse the chicks that have performed the replication operation to any position in the search space according to a certain probability. Through this operation, the chicken swarm can avoid falling into the local extrema. The specific reproduction and elimination-dispersal operations are as follows:

#### 3.1.1. Reproduction Operation

According to the fitness function values of the chicken swarm, let the chicks with poor optimization ability inherit the position of the chickens with the strongest optimization ability. The formula is as follows:

(7) $$\begin{array}{c} X_{i,j}\left(t+1\right)=X_{i-r\text{Num}-h\text{Num},j}\left(t\right), \end{array}$$

where *rNum* is the number of roosters and *hNum* is the number of hens.

#### 3.1.2. Elimination-Dispersal Operation

The chicks are dispersed to any position in the search space with the probability *P*_*ed*_, where *P*_*ed*_=0.25. The concrete contents are given as follows:

for *i* = (*rNum* + *hNum* + 1): *pop* do.
 if *p* > rand then
  (8) $$\begin{array}{c} X_{i,j}\left(t+1\right)=lb+\left(ub-lb\right)\times \text{rand}. \end{array}$$
 end.
end.

Here, *pop* is the population size. *lb* and *ub* are the lower and upper bounds of search range, respectively.

### 3.2. CSO Algorithm Based on PSO (CSO-PSO Algorithm)

To improve the global optimization ability of the CSO algorithm, in this section, we construct a CSO-PSO algorithm to enhance the ability of the algorithm to jump out of the local extrema by integrating PSO into the CSO algorithm. The flowchart of the CSO-PSO algorithm is shown in Figure 2.

The main steps are described as follows:

1. *Population initialization.* It mainly involves the parameter settings and determination of initial individual between CSO and PSO algorithms.
2. *Fitness evaluation.* The initial swarm optimal value is recorded on the bulletin board.
3. *Subgroup division.* The initial population is divided into two parts with the same scale as follows: subgroup 1 and subgroup 2.
4. *CSO.* We assign roles to subgroup 1 according to the CSO algorithm and perform the foraging behavior of the chicken swarm to search for the global optimal value.
5. *PSO.* The velocity and position of particles in subgroup 2 are updated according to the PSO algorithm to search for the global optimal value.
6. *Information exchange.* We merge subgroup 1 and subgroup 2 to realize information exchange.
7. *Updating swarm optimal value.* The swarm optimal value is updated according to the subgroup optimal values obtained in steps (4) and (5).
8. Werepeat steps (3)–(7) until the maximum number of iterations is reached and the optimal value is output.

### 3.3. ICSO Algorithm

In view of the premature convergence problem of the standard CSO algorithm in dealing with multimodal optimization problems, an ICSO algorithm is proposed in this section. Considering that the chicks have the weakest optimization ability in the whole chicken swarm, the RECSO algorithm in Section 3.1 is introduced to improve the depth search ability of the algorithm. At the same time, the CSO-PSO algorithm in Section 3.2 is introduced to improve the global search ability of the algorithm. The flowchart of the ICSO algorithm is shown in Figure 3. The green part is the improvement strategy of reproduction and elimination-dispersal operations introduced in Section 3.1 and the yellow part is the improvement strategy of the PSO algorithm integrated in Section 3.2.

The corresponding detailed steps are as follows:

(1) *Parameter settings.* It mainly involves the maximum number of iterations *M*, the population size *pop*, the dimension of solution space *dim*, and the limited number of role updates *G.*
(2) *Population initialization. pop* solutions are randomly generated in the solution space of the optimization problem, which are used as the initial positions of the population. According to the fitness function of the optimization problem, the fitness value of each position is calculated as a food source.
(3) *Fitness evaluation.* By comparing the food source content of the whole initial population, the optimal food source and corresponding individual position of the population are recorded.
(4) *Subgroup division.* The whole population is randomly divided into two parts, namely, subgroup 1 and subgroup 2.
(5) *RECSO.* The subgroup 1 is optimized according to the RECSO algorithm. The details are summarized as follows:
  - *Judgment of the role update condition.* The role update condition of the whole algorithm is mod*(t*,*G)* = = 1, where *t* is the current iteration number, mod is a remainder function. If the condition is false, we jump to step (d); otherwise, we judge whether it is the first iteration of the algorithm, if so, we go to step (c), if not, we go to step (b).
  - *Reproduction and elimination-dispersal operations.* We perform the reproduction and elimination-dispersal operations which are described in Section 3.1 on the chicks.
  - *Role assignment and subgroup division.* According to the fitness function of the current chicken swarm, we update the hierarchical order and mother-child relationship of the whole chicken swarm. After that, we divide the subgroups and determine the number of subgroups according to the number of the roosters. Each rooster belongs to different subgroups. The hens and chicks are randomly assigned to different subgroups, but it is necessary to ensure that there is at least one hen in each subgroup.
  - *Foraging behavior.* According to (1), (3), and (6), the foraging behaviors are performed by chickens with different roles.
  - *Update of the optimal food source.* At the end of each iteration, the optimization situation of chickens with different roles will change accordingly. We calculate the food source content of the current chicken swarm according to the fitness function and record the optimal food source and its corresponding position by comparing them with the previous situation.
(6) *PSO.* The velocity and position of particles in subgroup 2 are updated according to the PSO algorithm. The optimal food source and its corresponding position are recorded.
(7) *Information interaction.* We merge subgroups 1 and 2 to realize the information interaction.
(8) *Update of swarm optimal value.* The swarm optimal value is updated according to the subgroup optimal values obtained in steps (e) and (6).
(9) *Judgment of the algorithm's termination conditions.* If the maximum number of iterations specified by the algorithm is reached, the optimal value is output and the program operation is ended; otherwise, we jump to step (4).

## 4. Simulation Experiment

### 4.1. Experimental Setup

#### 4.1.1. The Experimental Environment

The experimental environment of this paper is described as follows: Windows 7 operating system, CPU: 3.5 GHz RAM: 12 GB and the programming environment is MATLAB R2016a. In order to verify the effectiveness and superiority of the ICSO algorithm, we conducted experiments on CEC2014 function test suite, which provides 30 test functions, including 3 unimodal functions: *f*_1_∼*f*_3_, 13 simple multimodal functions: *f*_4_∼*f*_16_, 6 hybrid functions: *f*_17_∼*f*_22_, and 8 composition functions: *f*_23_∼*f*_30_. The search range of all test functions is [−100 100]. In order to understand CEC2014 function test suite more intuitively, the function types, numbers, names, and theoretical global optimal values are given in Table 1.

#### 4.1.2. The Parameter Settings

To make a more reasonable comparison, for all algorithms involved in this paper, the population size is set to 100, the maximum number of iterations is 10000, and the dimension of solution space is 10. All algorithms are independently run 30 times on each test function, and then the mean values are calculated. Other parameter settings involved in this experiment are as follows:

1. *Parameter settings of ICSO and CSO algorithms.* The limited number of role updates in the chicken swarm *G* = 10. The ratios of roosters and hens in the whole chicken swarm *rPercent* and *hPercent* are 0.15 and 0.7, respectively. The proportion of mother hens in the hens *mPercent* = 0.5. In addition, the elimination-dispersal probability *P*_*ed*_ of the ICSO algorithm is 0.25.
2. *Parameter settings of BFA.* The chemotactic operation *Nc* = 100. The reproduction operation *Nre* = 10. The elimination-dispersal operation *N*_*ed*_ = 10, and the length of a swim *Ns* = 4.
3. *Parameter settings of the PSO algorithm.* Two learning factors *c*_1_ and *c*_2_ are both 2.
4. *Parameter settings of AFSA.* The visual field of artificial fish visual = 2.5. The step length step = 0.3. The maximum tentative number try_number = 5.
5. *Parameter settings of GA.* The binary digits *PRECI* = 20. The generation gap *GGAP* = 0.9. The crossover probability *P*_*c*_ = 0.7, and the mutation probability *P*_*m*_ = 0.01.

In aforementioned parameter settings, the parameters of CSO, BFA, and AFSA are set according to the literature [13, 25] and [14], where CSO, BFA, and AFSA are proposed. It is worth noting that the reason why *N*_*re*_ and *N*_*ed*_ are set to 10 in BFA is to ensure that the maximum number of iterations is 10000. The parameter settings of PSO and GA are derived from the comparison algorithms mentioned in the literature [28, 32], respectively.

In the ICSO algorithm, considering that if the value of *P*_*ed*_ is large, chicks are easy to fall into random exhaustive search. If the value of *P*_*ed*_ is small, it is not conducive to maintaining population diversity, which will reduce the local search ability of the algorithm. Therefore, in this section, to give an appropriate value of *P*_*ed*_, we select four typical functions *f*_3_, *f*_6_, *f*_20_, and *f*_27_ from the CEC2014 function test suite for experiments, where *f*_3_ is a unimodal function, *f*_6_ is a simple multimodal function, *f*_20_ is a hybrid function, and *f*_27_ is a composition function. At the same time, we choose the ICSO algorithm to run these four functions 30 times independently to calculate their mean values. The experimental results are shown in Table 2.

In Table 2, *F*_i_^*∗*^ represents the theoretical global optimal values corresponding to different functions, where *i* = 3, 6, 20, 27. The value of *P*_*ed*_ is taken from 0.05 to 0.85 with an interval of 0.2. |*D*_i_| represents the absolute value of the difference between the theoretical global optimal value and the actual mean one obtained on each function, where *i* = 0.05, 0.25, ⋯, 0.85. It is easy to see from Table 2 that when *P*_*ed*_ = 0.25, the value of |*D*_i_| is the smallest, that is, the actual mean optimal values obtained by the ICSO algorithm on four functions are the closest to the theoretical ones. Furthermore, when the value of *P*_*ed*_ changes from 0.25 to 0.85 with an interval of 0.2, the value of |*D*_i_| is larger than that of |*D*_0.25_|. Therefore, in the experiment, we choose *P*_*ed*_ = 0.25.

### 4.2. The Effectiveness Test of ICSO, RECSO, and CSO-PSO

To verify the effectiveness of the three improved algorithms proposed in this paper, namely ICSO, RECSO, and CSO–PSO, compared with the standard CSO algorithm, in this section, these four algorithms are tested on the CEC2014 function test suite, and the experimental comparison is made in terms of optimization accuracy and convergence performance. The experimental parameter settings are shown in Section 4.1.

#### 4.2.1. The Effectiveness Test for Optimization Accuracy

To verify the effectiveness of the three improved algorithms (ICSO, RECSO, and CSO-PSO) in terms of optimization accuracy, in this section, we use ICSO, RECSO, CSO-PSO, and CSO to run all 30 functions of the CEC2014 test suite independently 30 times to obtain their mean values. The results are shown in Table 3, where the symbols “>,” “=,” and “<” indicate that the experimental results of the comparison algorithms are superior, equal, and inferior to the CSO algorithm, respectively. The optimal results are shown in bold.

It can be clearly seen from Table 3 that the ICSO algorithm has the largest number of optimal values, followed by CSO-PSO, and the CSO algorithm is the worst. Most specifically, the operation results of the ICSO algorithm on 28 functions are better than those of the CSO algorithm, and the operation results on 2 functions are the same as those of the CSO algorithm. The operation results of the RECSO algorithm on 19 functions are better than those of the CSO algorithm. The operation results of it on 6 functions are worse than those of the CSO algorithm, and its operation results are the same as those of the CSO algorithm on the other 5 functions. The results of the CSO-PSO algorithm are similar to those of the ICSO algorithm. There are 28 functions whose operation results are better than those of the CSO algorithm, and the operation results on 2 functions are the same as those of the CSO algorithm. However, from the number of optimal values obtained, the ICSO algorithm is far superior to the CSO-PSO algorithm. This shows the effectiveness of the three improved strategies in terms of optimization accuracy compared with the CSO algorithm, and the performance of the ICSO algorithm is the best among the four algorithms.

#### 4.2.2. The Effectiveness Test for Convergence Performance

To verify the effectiveness of the abovementioned three improved algorithms in terms of convergence performance compared to the CSO algorithm, Figure 4 shows the average convergence curves of the four algorithms independently running 30 times on 30 functions. In order to show the convergence effect of each algorithm more clearly, the average fitness function values are logarithmically processed in Figure 4. In addition, the convergence curves of some functions contain subgraphs, such as those of *f*_4_, *f*_8_, and *f*_13_, which are locally magnified renderings.

It can be seen from Figure 4 that the convergence performance of the ICSO algorithm on functions *f*_1_, *f*_5_, *f*_9_, *f*_10_, *f*_11_, *f*_17_, *f*_18_, *f*_25_, and *f*_27_ is significantly better than that of the other three algorithms. On functions *f*_2_, *f*_3_, *f*_6_, *f*_8_, *f*_12_, *f*_16_, *f*_22_, and *f*_24_, ICSO and CSO-PSO algorithms have similar convergence performance. The former is slightly better than the latter, and both of them are better than CSO and RECSO algorithms (only on function *f*_16_, CSO-PSO algorithm is slightly better than the ICSO algorithm). On functions *f*_4_, *f*_7_, *f*_13_, *f*_14_, *f*_15_, *f*_19_, *f*_20_, *f*_21_, *f*_28_, *f*_29_, and *f*_30_, the four algorithms have comparable convergence performance, and ICSO is slightly superior. On functions *f*_23_ and *f*_26_, the RECSO algorithm has the best convergence performance.

To sum up, the convergence performance of the ICSO algorithm on 27 functions is the best, and it is better than that of the CSO algorithm on all 30 functions. The CSO-PSO algorithm has the best convergence performance on one function, and its convergence performance on 28 functions is better than that of the CSO algorithm. The RECSO algorithm has the best convergence performance on two functions, and only the convergence performance on functions *f*_8_, *f*_13_, and *f*_17_ is slightly inferior to that of the CSO algorithm. This fully shows the effectiveness of the three improved algorithms in terms of convergence performance compared with the CSO algorithm, and the ICSO algorithm has the best convergence performance.

It is concluded that the reason why the ICSO algorithm is superior to the other three algorithms may be that the algorithm integrates the ideas of BFA and PSO, which not only improves the depth search ability of the algorithm but also improves its breadth searchability.

### 4.3. The Superiority Comparison among Several Swarm Intelligent Algorithms

To verify the superiority of the ICSO algorithm proposed in this paper, in this section, we compare the performance of seven algorithms, namely, ICSO, CSO, ICSOII proposed in the literature [30] (named ICSOII to distinguish it from the ICSO algorithm), BFA, PSO, AFSA, and GA from the aspects of optimization accuracy and convergence performance.

#### 4.3.1. The Superiority Comparison in Optimization Accuracy

To verify the superiority of the ICSO algorithm in terms of optimization accuracy, this section presents the experimental results of the abovemetioned seven algorithms to optimize the CEC2014 function test suite. The data in Table 4 are the mean values of 30 independent runs of each algorithm on each function. The bold data in Table 4 are the optimal values.

It can be seen from Table 4 that for functions *f*_1_ and *f*_2_, the ICSO algorithm directly reduces the order of magnitude of optimization accuracy from 5 and 7 to 3 and 2, respectively. In addition, from the number of optimal values that can be found, the number of optimal values that can be found by CSO and GA is 2. AFSA and PSO can find 3 and 9 optimal values, respectively. The optimal value of ICSOII and BFA is both 6. The number of optimal values that can be found by the ICSO algorithm is 18, which shows the superiority of the ICSO algorithm in optimization accuracy.

#### 4.3.2. The Superiority Comparison in Convergence Performance

To verify the superiority of the ICSO algorithm in convergence performance, in this section, we give the average convergence curves of 30 test functions on the CEC2014 function test suite optimized by the abovementioned seven algorithms (each algorithm is independently run 30 times on each test function). The parameter settings in this section are shown in Section 4.1.2. As mentioned in Section 4.2.2, the ordinates in Figure 5 are the logarithms of the average fitness function values, and subgraphs in some convergence curves are locally magnified renderings, so as to show the convergence effect of each algorithm more clearly.

It can be seen from Figure 5 that the convergence performance of the ICSO algorithm is the best on functions *f*_1_, *f*_5_∼*f*_7_, *f*_11_, *f*_14_, *f*_15_, *f*_17_, *f*_19_, *f*_21_, *f*_22_, *f*_24_, *f*_25_, and *f*_27_, among which, on the functions *f*_5_, *f*_6_, *f*_11_, *f*_25_, and *f*_27_, the convergence advantage of the ICSO algorithm is particularly obvious. On functions *f*_2_, *f*_3_, *f*_8_, *f*_9_, and *f*_20_, the convergence performance between ICSO and PSO algorithms is very close, the performance of the PSO algorithm is slightly better, and they all outperform the performance of the other algorithms. On functions *f*_13_ and *f*_26_, the convergence performance of ICSO and CSO algorithms is the best, and the performance of the ICSO algorithm is slightly inferior to that of the CSO algorithm, ranking second. On the function *f*_16_, ICSOII has the best convergence performance and the ICSO algorithm ranks second. Only on functions *f*_4_, *f*_12_, *f*_18_, *f*_23_, and *f*_28_∼*f*_30_, the convergence performance of the ICSO algorithm is not as good as that of BFA, AFSA, and GA, ranking 3^rd^ or 4^th^. From this, we can see the superiority of the ICSO algorithm proposed in this paper in terms of convergence performance.

#### 4.3.3. Friedman Test of Algorithms

To compare the performance of various algorithms more reasonably, this section uses the Friedman test to test the performance of the abovementioned 7 algorithms (ICSO, ICSOII, PSO, CSO, GA, BFA, and AFSA) from a statistical point of view. The Friedman test is a nonparametric test method, which is often used to test the performance of algorithms due to its simple operation and lax requirements on the test data [32, 33, 36]. For the minimum optimization problem, the smaller the average ranking of the algorithm, the better its performance.  Table 5 is the Friedman test results of 7 algorithms on 30 functions.

It can be seen from Table 5 that the average ranking of the ICSO algorithm is 1.90, ranking the highest, 0.87 lower than that of ICSOII, 2.70 lower than that of the CSO algorithm and 1.38 lower than that of the PSO algorithm, which fully demonstrates the effectiveness of the improved strategy in this paper.

To sum up, the reason why the ICSO algorithm is superior to CSO, PSO, and BFA may be that it greatly enhances the ability of the algorithm to jump out of the local extrema by innovative cooperation between the chicken swarm and particle one to achieve information interaction and improves the depth searchability of the algorithm by integrating the replication and elimination-dispersal operations of BFA. The reason why the ICSO algorithm is superior to ICSOII, GA, and AFSA may be that the ICSO algorithm has a mechanism of subgroup division and multiswarm cooperation based on chicken swarm and particle one, which realizes parallel optimization through group cooperation. Although the ICSOII algorithm has subgroup division, its population cooperation is limited to the cooperation within the chicken swarm, so its optimization ability is weaker than that of the ICSO algorithm.

### 4.4. Experimental Comparison between ICSO and ICSOII

To further compare the performance between the ICSO algorithm proposed in this paper and the ICSOII algorithm proposed in the literature [30], we set the parameters of the algorithm according to the literature [30] in this section. The statistical results of the abovementioned two algorithms running 51 times independently on the CEC2014 function test suite are shown in Table 6. The experimental data of the ICSOII algorithm comes from its corresponding literature.

It can be clearly seen from Table 6 that the number of optimal values obtained by the ICSOII algorithm is 18, and the theoretical optimal values are obtained on 10 functions. While the number of optimal values obtained by the ICSO algorithm is 21, and its theoretical optimal values are obtained on 12 functions.

### 4.5. Experimental Comparison between ICSO and a State-of-the-Art Algorithm

To further verify the performance of the ICSO algorithm, DMSDL-QBSA which is a state-of-the-art algorithm proposed in the literature [18] is also used to compare with the ICSO algorithm in this section. In order to make the experimental comparison fairer and more reasonable, the parameter settings of the ICSO algorithm are the same as those of DMSDL-QBSA, that is, the population size is set to 30, and the maximum number of iterations is set to 100000. Other parameter settings can be seen in Section 4.1.2.

The experimental data including the maximum (Max), minimum (Min), mean (Mean), and variance (Var) values are shown in Table 7, where the optimal results are shown in bold. It is worth noting that the experimental data of DMSDL-QBSA are extracted from its corresponding literature.

By analyzing the data in Table 7, we can see that our ICSO algorithm can get all the best values on functions *f*_1_∼*f*_3_, *f*_5_∼*f*_9_, *f*_12_∼*f*_21_, *f*_26_, and *f*_29_. On functions *f*_4_, *f*_11_, *f*_22_, *f*_24_, *f*_25_, and *f*_30_, the ICSO algorithm has the best results in terms of the maximum, minimum, and mean values but is slightly inferior to DMSDL-QBSA in variance value. DMSDL-QBSA only achieves relatively good results on functions *f*_23_, *f*_27_, and *f*_28_. To sum up, our ICSO algorithm has advantages in most test functions due to the improvement of global and deep search abilities.

### 4.6. Welded Beam Design Problem

To verify the performance of the ICSO algorithm to solve practical optimization problems, a welded beam design problem is considered, which has been described in detail in the literature [4, 37] and [38]. The problem is a minimum problem, which can be formulated as follows:

(9) $$\begin{array}{c} \text{Minimize}f\left(x\right)=1.10471x_{1}^{2}x_{2}+0.04811x_{3}x_{4}\left(14.0+x_{2}\right),\\ \text{Subject to}g_{1}\left(x\right)=\tau \left(x\right)-\tau_{\text{max}}\leq 0,\\ g_{2}\left(x\right)=\sigma \left(x\right)-\sigma_{\text{max}}\leq 0,\\ g_{3}\left(x\right)=x_{1}-x_{4}\leq 0,\\ g_{4}\left(x\right)=0.10471x_{1}^{2}+0.04811x_{3}x_{4}\left(14.0+x_{2}\right)-5.0\leq 0,\\ g_{5}\left(x\right)=0.125-x_{1}\leq 0,\\ g_{6}\left(x\right)=\delta \left(x\right)-\delta_{\text{max}}\leq 0,\\ g_{7}\left(x\right)=P-P_{c}\left(x\right)\leq 0, \end{array}$$

where 0.1 ≤ *x*_1_, *x*_4_ ≤ 2, 0.1 ≤ *x*_2_, *x*_3_ ≤ 10,

(10) $$\begin{array}{c} \tau \left(x\right)=\sqrt{{\left({\left(\tau '\right)}^{2}+2\tau '\tau^{\prime \prime }\frac{x_{2}}{2R}+\left(\tau “\right)\right)}^{2}},\tau '=\frac{P}{\sqrt{2}x_{1}x_{2}},\tau^{\prime \prime }=\frac{MR}{J},\\ M=P\left(L+\frac{x_{2}}{2}\right),R=\sqrt{\frac{x_{2}^{2}}{4}+{\left(\frac{x_{1}+x_{3}}{2}\right)}^{2}},\\ J=2\left\{\sqrt{2}x_{1}x_{2}\left[\frac{x_{2}^{2}}{12}+{\left(\frac{x_{1}+x_{3}}{2}\right)}^{2}\right]\right\},\sigma \left(x\right)=\frac{6PL}{x_{4}x_{3}^{2}},\delta \left(x\right)=\frac{4PL^{3}}{Ex_{4}x_{3}^{3}},\\ P_{c}\left(x\right)=\frac{4.013E\sqrt{x_{4}^{6}x_{3}^{2}/36}}{L^{2}}\left(1-\frac{x_{3}}{2L}\sqrt{\frac{E}{4G}}\right). \end{array}$$

*P*=6000*lb*, *L* = 14in., *E* = 30 × 10^6^ psi, *G* = 12 × 10^6^ psi, *τ*_max_ = 13600 psi, *σ*_max_ = 30000, *δ*_max_=0.25 in.

The comparison results of optimal solutions obtained by different algorithms are shown in Table 8. The statistical results are shown in Table 9, where “Worst,” “Mean,” “Best,” and “SD” stand for the worst, mean, best, and standard deviation values obtained by 30 independent runs, respectively. In addition, the optimal results are shown in bold. It is worth noting that the experimental results of comparison algorithms are extracted from their corresponding literature.

For HFPSO [4] and EPSO [37], because the optimal solutions of the four parameters are not given in the literature [4, 37], they are not listed in Table 8. It can be seen from Tables 8 and 9, ICSO and MBA [38] have obvious advantages over the other two algorithms in terms of the worst, mean values, standard deviation, etc. Although the stability of the ICSO algorithm is slightly inferior to that of MBA [38], it has a higher optimization accuracy, which preliminarily shows that ICSO can be used to solve the welded beam design problem.

## 5. Conclusion and Future Directions

To overcome the premature convergence problem of the standard CSO algorithm when solving complex optimization problems, an ICSO algorithm is proposed in this paper. For the chicks with the weakest optimization ability, we introduce the reproduction and elimination-dispersal operations of BFA to improve the deep searchability of the CSO algorithm. In addition, in order to improve the global convergence speed of the algorithm, the theory of PSO is integrated to construct a hybrid CSO algorithm. The experimental results show that the ICSO algorithm proposed in this paper can significantly improve the optimization accuracy and convergence performance.

The disadvantage of the proposed algorithm is that with the increase of the dimension of the optimization problem, the optimization ability of the algorithm will decrease, which makes it not suitable for dealing with large-scale optimization problems. Therefore, in the future research work, how to dynamically adjust the limited number of role updates in the chicken swarm according to the number of iterations and how to improve the individual position update formula for hens with relatively weak search ability to further improve the optimization ability still need further research. In addition, we will also consider applying the ICSO algorithm to deal with practical problems, such as path planning in logistics distribution, workshop scheduling, and land use forecast [39].

## Figures and Tables

**Figure 1:** Flowchart of the standard CSO algorithm.

**Figure 2:** Flowchart of CSO-PSO algorithm.

**Figure 3:** Flowchart of ICSO algorithm.

**Figure 4:** Convergence curves of 4 algorithms on 30 test functions.

**Figure 5:** Convergence curves of 7 algorithms on 30 test functions.

**Table 1:** The description of the CEC2014 test functions.

Type	No	Functions	*F*_i_^*∗*^
Unimodal functions	*f*_1_	Rotated high conditioned elliptic function	100
	*f*_2_	Rotated bent cigar function	200
	*f*_3_	Rotated discus function	300

Simple multimodal functions	*f*_4_	Shifted and rotated Rosenbrock's function	400
	*f*_5_	Shifted and rotated Ackley's function	500
	*f*_6_	Shifted and rotated Weierstrass's function	600
	*f*_7_	Shifted and rotated Griewank's function	700
	*f*_8_	Shifted Rastrigin's function	800
	*f*_9_	Shifted and rotated Rastrigin's function	900
	*f*_10_	Shifted Schwefel's function	1000
	*f*_11_	Shifted and rotated Schwefel's function	1100
	*f*_12_	Shifted and rotated katsuura function	1200
	*f*_13_	Shifted and rotated HappyCat function	1300
	*f*_14_	Shifted and rotated HGBat function	1400
	*f*_15_	Shifted and rotated expanded Griewank's plus Rosenbrock's function	1500
	*f*_16_	Shifted and rotated expanded Scaffer's F6 function	1600

Hybrid functions	*f*_17_	Hybrid function 1 (*N* *=* 3)	1700
	*f*_18_	Hybrid function 2 (*N* *=* 3)	1800
	*f*_19_	Hybrid function 3 (*N* *=* 4)	1900
	*f*_20_	Hybrid function 4 (*N* *=* 4)	2000
	*f*_21_	Hybrid function 5 (*N* *=* 5)	2100
	*f*_22_	Hybrid function 6 (*N* *=* 5)	2200

Composition functions	*f*_23_	Composition function 1 (*N* *=* 5)	2300
	*f*_24_	Composition function 2 (*N* *=* 3)	2400
	*f*_25_	Composition function 3 (*N* *=* 3)	2500
	*f*_26_	Composition function 4 (*N* *=* 5)	2600
	*f*_27_	Composition function 5 (*N* *=* 5)	2700
	*f*_28_	Composition function 6 (*N* *=* 5)	2800
	*f*_29_	Composition function 7 (*N* *=* 3)	2900
	*f*_30_	Composition function 8 (*N* *=* 3)	3000

**Table 2:** The experimental results via different *P*_*ed*_.

Functions	*f*_3_	*f*_6_	*f*_20_	*f*_27_
*F*_i_^*∗*^	300	600	2000	2700
*P*_*ed*_ = 0.05	300.1282	600.7110	2.0077*e + *03	2.8786*e + *03
|*D*_0.05_|	0.1282	0.7110	7.7	178.6
*P*_*ed*_ = 0.25	**300.0813**	**600.7149**	**2.0053*e + *03**	**2.8314*e + *03**
|*D*_0.25_|	0.0813	0.7149	5.3	131.4
*P*_*ed*_ = 0.45	300.1122	600.8051	2.0068*e + *03	2.8911*e + *03
|*D*_0.45_|	0.1122	0.8051	6.8	191.1
*P*_*ed*_ = 0.65	300.1803	600.8868	2.0075*e + *03	2.8463*e + *03
|*D*_0.65_|	0.1803	0.8868	7.5	146.3
*P*_*ed*_ = 0.85	300.1330	601.0191	2.0074*e + *03	2.8795*e + *03
|*D*_0.85_|	0.1330	1.0191	7.4	179.5

**Table 3:** The experimental results of ICSO, RECSO, CSO-PSO, and CSO algorithms.

Functions	ICSO	CSO	RECSO	CSO-PSO
*f*_1_	**2.5963*e + *03**>	7.4764*e + *05	3.2289*e + *05>	6.1321*e + *03>
*f*_2_	**728.1158**>	1.5107*e + *07	5.8310*e + *06>	1.0100*e + *03>
*f*_3_	**300.0813**>	957.7185	446.6751>	300.2133>
*f*_4_	**411.1957**>	431.2580	426.6130>	414.4211>
*f*_5_	**517.9530**>	519.9147	519.2104>	519.1367>
*f*_6_	**600.7149**>	602.1075	601.8348>	600.8712>
*f*_7_	**700.0947**>	701.4794	701.4910<	700.1054>
*f*_8_	**800.1327**>	808.6386	809.2422<	800.3648>
*f*_9_	**904.7067**>	911.8049	911.5464>	905.7708>
*f*_10_	**1.0499*e + *03**>	1.1771*e + *03	1.1783*e + *03<	1.1091*e + *03>
*f*_11_	**1.2233*e + *03**>	1.4489*e + *03	1.4199*e + *03>	1.2716*e + *03>
*f*_12_	**1.2001*e + *03**>	1.2005*e + *03	1.2005*e + *03=	**1.2001*e + *03**>
*f*_13_	**1.3001*e + *03=**	**1.3001*e + *03**	**1.3001*e + *03=**	**1.3001*e + *03=**
*f*_14_	**1.4001*e + *03**>	1.4003*e + *03	1.4003*e + *03=	**1.4001*e + *03**>
*f*_15_	**1.5007*e + *03**>	1.5011*e + *03	1.5009*e + *03>	1.5009*e + *03>
*f*_16_	**1.6015*e + *03**>	1.6020*e + *03	1.6020*e + *03=	**1.6015*e + *03**>
*f*_17_	**2.6873*e + *03**>	3.6491*e + *03	5.8702*e + *03<	3.0513*e + *03>
*f*_18_	**2.6243*e + *03**>	5.1907*e + *03	3.5783*e + *03>	4.7507*e + *03>
*f*_19_	**1.9008*e + *03**>	1.9023*e + *03	1.9018*e + *03>	1.9013*e + *03>
*f*_20_	**2.0053*e + *03**>	2.0848*e + *03	2.0673*e + *03>	2.0068*e + *03>
*f*_21_	**2.1390*e + *03**>	2.3364*e + *03	2.3150*e + *03>	2.1486*e + *03>
*f*_22_	**2.2045*e + *03**>	2.2244*e + *03	2.2264*e + *03<	2.2084*e + *03>
*f*_23_	2.6122*e + *03>	2.6138*e + *03	**2.5955*e + *03**>	2.6122*e + *03>
*f*_24_	**2.5148*e + *03**>	2.5258*e + *03	2.5211*e + *03>	2.5158*e + *03>
*f*_25_	**2.6629*e + *03**>	2.6923*e + *03	2.6713*e + *03>	2.6694*e + *03>
*f*_26_	**2.7001*e + *03=**	**2.7001*e + *03**	**2.7001*e + *03**=	**2.7001*e + *03=**
*f*_27_	**2.8314*e + *03**>	2.9131*e + *03	2.8878*e + *03>	2.8759*e + *03>
*f*_28_	**3.1761*e + *03**>	3.1878*e + *03	3.1792*e + *03>	3.1765*e + *03>
*f*_29_	**3.2961*e + *03**>	3.5482*e + *03	3.5628*e + *03<	3.3786*e + *03>
*f*_30_	**3.5856*e + *03**>	3.8147*e + *03	3.6982*e + *03>	3.7041*e + *03>
>	28	—	19	28
<	0	—	6	0
=	2	—	5	2
The number of optimal values	29	2	3	5

**Table 4:** The optimization accuracy comparison of 7 intelligent algorithms.

Function	ICSO	CSO	ICSOII	BFA	PSO	AFSA	GA
*f*_1_	**2.5963*e + *03**	7.4764*e + *05	2.6050*e + *05	7.8186*e + *05	3.0053*e + *03	3.4393*e + *06	4.4127*e + *04
*f*_2_	728.1158	1.5107*e + *07	1.0659*e + *03	8.9827*e + *03	**599.1427**	4.3975*e + *08	3.9775*e + *03
*f*_3_	300.0813	957.7185	857.3808	1.5267*e + *04	**300.0106**	1.7089*e + *03	3.3396*e + *03
*f*_4_	411.1957	431.2580	409.3101	**404.7945**	418.4158	499.9456	410.1793
*f*_5_	**517.9530**	519.9147	519.5907	520.0342	520.1769	520.1581	519.9999
*f*_6_	**600.7149**	602.1075	600.9178	609.8307	601.0835	609.2003	602.9651
*f*_7_	**700.0947**	701.4794	700.3004	700.3424	700.0974	722.0824	700.2899
*f*_8_	800.1327	808.6386	800.5306	847.2295	**800.0663**	842.1636	802.7196
*f*_9_	904.7067	911.8049	905.7401	951.4788	**904.5150**	932.2919	915.1409
*f*_10_	1.0499*e + *03	1.1771*e + *03	1.0717*e + *03	1.8578*e + *03	1.0897*e + *03	2.1799*e + *03	**1.0321*e + *03**
*f*_11_	**1.2233*e + *03**	1.4489*e + *03	1.2524*e + *03	2.0745*e + *03	1.2969*e + *03	2.2376*e + *03	1.6340*e + *03
*f*_12_	**1.2001*e + *03**	1.2005*e + *03	**1.2001*e + *03**	**1.2001*e + *03**	1.2002*e + *03	1.2005*e + *03	**1.2001*e + *03**
*f*_13_	**1.3001*e + *03**	**1.3001*e + *03**	**1.3001*e + *03**	1.3002*e + *03	**1.3001*e + *03**	1.3007*e + *03	1.3004*e + *03
*f*_14_	**1.4001*e + *03**	1.4003*e + *03	**1.4001*e + *03**	1.4003*e + *03	**1.4001*e + *03**	1.4006*e + *03	1.4004*e + *03
*f*_15_	**1.5007*e + *03**	1.5011*e + *03	1.5008*e + *03	1.5083*e + *03	1.5009*e + *03	1.5398*e + *03	1.5021*e + *03
*f*_16_	**1.6015*e + *03**	1.6020*e + *03	**1.6015*e + *03**	1.6038*e + *03	**1.6015*e + *03**	1.6035*e + *03	1.6027*e + *03
*f*_17_	**2.6873*e + *03**	3.6491*e + *03	3.1426*e + *03	9.7385*e + *03	3.1797*e + *03	2.8286*e + *03	3.5779*e + *04
*f*_18_	2.6243*e + *03	5.1907*e + *03	2.1108*e + *03	7.3224*e + *03	4.7427*e + *03	**1.9077*e + *03**	1.4040*e + *04
*f*_19_	**1.9008*e + *03**	1.9023*e + *03	**1.9008*e + *03**	1.9222*e + *03	1.9013*e + *03	1.9092*e + *03	1.9014*e + *03
*f*_20_	2.0053*e + *03	2.0848*e + *03	2.0067*e + *03	6.8899*e + *03	**2.0040*e + *03**	2.1115*e + *03	8.6438*e + *03
*f*_21_	**2.1390*e + *03**	2.3364*e + *03	2.1546*e + *03	5.9637*e + *03	2.1501*e + *03	2.5022*e + *03	5.3393*e + *03
*f*_22_	**2.2045*e + *03**	2.2244*e + *03	2.2063*e + *03	2.4322*e + *03	2.2077*e + *03	2.2462*e + *03	2.2689*e + *03
*f*_23_	2.6122*e + *03	2.6138*e + *03	2.5766*e + *03	**2.5000*e + *03**	2.6295*e + *03	**2.5000*e + *03**	2.6295*e + *03
*f*_24_	**2.5148*e + *03**	2.5258*e + *03	2.5159*e + *03	2.5769*e + *03	2.5153*e + *03	2.5745*e + *03	2.5312*e + *03
*f*_25_	**2.6629*e + *03**	2.6923*e + *03	2.6766*e + *03	2.6965*e + *03	2.6871*e + *03	2.6952*e + *03	2.6890*e + *03
*f*_26_	**2.7001*e + *03**	**2.7001*e + *03**	**2.7001*e + *03**	2.7002*e + *03	**2.7001*e + *03**	2.7007*e + *03	2.7003*e + *03
*f*_27_	**2.8314*e + *03**	2.9131*e + *03	2.9066*e + *03	2.8737*e + *03	2.9798*e + *03	2.8807*e + *03	3.0434*e + *03
*f*_28_	3.1761*e + *03	3.1878*e + *03	3.1799*e + *03	**3.0000*e + *03**	3.2304*e + *03	**3.0000*e + *03**	3.2409*e + *03
*f*_29_	3.2961*e + *03	3.5482*e + *03	3.3122*e + *03	**3.1000*e + *03**	1.1433*e + *05	3.1064*e + *03	1.1836*e + *05
*f*_30_	3.5856*e + *03	3.8147*e + *03	3.6306*e + *03	**3.2000*e + *03**	3.6875*e + *03	3.2197*e + *03	3.8617*e + *03
The number of optimal values	18	2	6	6	9	3	2

**Table 5:** Friedman test results of 7 algorithms.

Algorithm	Average ranking	Ranking
ICSO	1.90	1
ICSOII	2.77	2
PSO	3.28	3
CSO	4.60	4
BFA	5.07	5
GA	5.13	6
AFSA	5.25	7

**Table 6:** The experimental results between ICSO and ICSOII.

Function	ICSO	ICSOII
*f*_1_	**3.74*e + *03** **±** **4.81*e ***±*** *03**	5.55*e + *04 ± 4.75*e **** ***±*** ***04
*f*_2_	**8.63*e + *02** **±** **5.85*e + *02**	1.08*e + *03 ± 2.71*e + *02
*f*_3_	**3.00*e + *02** **±** **1.19*e − *01**	7.71*e + *02 ± 2.86*e + *02
*f*_4_	4.14*e + *02 ± 1.45*e + *01	**4.00*e + *02** **±** **1.88*e − *01**
*f*_5_	**5.18*e + *02** **±** **4.75*e + *00**	5.19*e + *02 ± 5.97*e + *00
*f*_6_	**6.00*e + *02** **±** **9.13*e − *01**	**6.00*e + *02** **±** **1.24*e + *00**
*f*_7_	**7.00*e + *02** **±** **4.93*e − *02**	**7.00*e + *02** **±** **1.00*e − *02**
*f*_8_	**8.00*e + *02** **±** **5.16*e − *01**	8.03*e + *02 ± 3.77*e + *00
*f*_9_	**9.05*e + *02** **±** **1.94*e + *00**	9.06*e + *02 ± 4.06*e + *00
*f*_10_	**1.05*e + *03** **±** **6.31*e + *01**	1.06*e + *03 ± 2.36*e + *02
*f*_11_	**1.25*e + *03** **±** **1.13*e + *02**	1.46*e + *03 ± 2.01*e + *02
*f*_12_	**1.20*e + *03** **±** **1.46*e − *01**	**1.20*e + *03** **±** **3.14*e − *02**
*f*_13_	**1.30*e + *03** **±** **2.95*e − *02**	**1.30*e + *03** **±** **6.97*e − *02**
*f*_14_	**1.40*e + *03** **±** **2.42*e − *02**	**1.40*e + *03** **±** **7.79*e − *02**
*f*_15_	**1.50*e + *03** **±** **2.56*e − *01**	**1.50*e + *03** **±** **1.81*e − *01**
*f*_16_	**1.60*e + *03** **±** **4.21*e − *01**	**1.60*e + *03** **±** **3.18*e − *01**
*f*_17_	2.83*e + *03 ± 7.98*e + *02	**2.16*e + *03** **±** **2.47*e + *02**
*f*_18_	3.07*e + *03 ± 1.78*e + *03	**1.91*e + *03** **±** **6.00*e + *01**
*f*_19_	**1.90*e + *03** **±** **7.00*e − *01**	**1.90*e + *03** **±** **3.48*e − *01**
*f*_20_	**2.00*e + *03** **±** **5.27*e + *00**	2.10*e + *03 ± 6.34*e + *01
*f*_21_	**2.12*e + *03** **±** **4.53*e + *01**	2.36*e + *03 ± 6.19*e + *00
*f*_22_	**2.20*e + *03** **±** **9.25*e + *00**	2.22*e + *03 ± 7.12*e + *01
*f*_23_	2.50*e + *03 ± 3.07*e + *01	**2.40*e + *03** **±** **7.12*e + *01**
*f*_24_	**2.51*e + *03** **±** **3.71*e + *00**	2.52*e + *03 ± 4.68*e + *00
*f*_25_	2.67*e + *03 ± 3.33*e + *01	**2.61*e + *03** **±** **9.46*e + *00**
*f*_26_	**2.70*e + *03** **±** **2.35*e − *02**	**2.70*e + *03** **±** **4.46*e − *02**
*f*_27_	2.84*e + *03 ± 1.67*e + *02	**2.70*e + *03** **±** **6.15*e + *01**
*f*_28_	3.17*e + *03 ± 4.05*e + *01	**3.00*e + *03** **±** **6.35*e + *01**
*f*_29_	3.26*e + *03 ± 9.56*e + *01	**3.14*e + *03** **±** **9.52*e + *01**
*f*_30_	3.60*e + *03 ± 8.94*e + *01	**3.47*e + *03** **±** **6.87*e + *01**
The number of optimal values	21	18

**Table 7:** The experimental results between ICSO and DMSDL-QBSA.

Function	Term	ICSO	DMSDL-QBSA
*f*_1_	Max	**1.2436*e + *03**	9.6209*e + *08
	Min	**102.9899**	1.7687*e + *05
	Mean	**447.9202**	1.9320*e + *06
	Var	**7.9873*e + *04**	1.3093*e + *07

*f*_2_	Max	**226.3723**	1.7326*e + *10
	Min	**200.0070**	1.4074*e + *05
	Mean	**206.8620**	4.8412*e + *07
	Var	**51.1127**	4.2984*e + *08

*f*_3_	Max	**300**	5.3828*e + *06
	Min	**300**	6.3986*e + *02
	Mean	**300**	3.0848*e + *03
	Var	**3.2679*e*** − **25**	8.0572*e + *04

*f*_4_	Max	**436.1827**	4.3338*e + *03
	Min	**400.0000**	4.1267*e + *02
	Mean	**406.3343**	4.3261*e + *02
	Var	153.6519	**8.5548*e + *01**

*f*_5_	Max	**520.2256**	5.2110*e + *02
	Min	**500**	5.2007*e + *02
	Mean	**518.7619**	5.2014*e + *02
	Var	26.0152	**9.9700*e*** − **02**

*f*_6_	Max	**603.1944**	6.1569*e + *02
	Min	**600**	6.0257*e + *02
	Mean	**601.0094**	6.0358*e + *02
	Var	**0.9590**	1.3117*e + *00

*f*_7_	Max	**700.3289**	9.3907*e + *02
	Min	**700.0246**	7.0069*e + *02
	Mean	**700.1142**	7.0290*e + *02
	Var	**0.0038**	1.3815*e + *01

*f*_8_	Max	**800.9950**	9.3391*e + *02
	Min	**800**	8.0877*e + *02
	Mean	**800.1327**	8.1676*e + *02
	Var	**0.1183**	9.7968*e + *00

*f*_9_	Max	**908.9546**	1.0366*e + *03
	Min	**900.9950**	9.1537*e + *02
	Mean	**904.9416**	9.2335*e + *02
	Var	**3.3100**	9.3860*e + *00

*f*_10_	Max	**1.2722*e + *03**	3.4795*e + *03
	Min	**1.0151*e + *03**	1.4316*e + *03
	Mean	**1.1078*e + *03**	1.6111*e + *03
	Var	8.5848*e + *03	**2.2195*e + *02**

*f*_11_	Max	**1.6046*e + *03**	3.7357*e + *03
	Min	**1.1119*e + *03**	1.2811*e + *03
	Mean	**1.2712*e + *03**	1.4869*e + *03
	Var	2.0085*e + *04	**2.6682*e + *02**

*f*_12_	Max	**1.2003*e + *03**	1.2044*e + *03
	Min	**1.2000*e + *03**	1.2017*e + *03
	Mean	**1.2001*e + *03**	1.2018*e + *03
	Var	**0.0062**	2.1603***e*** − 01

*f*_13_	Max	**1.3001*e + *03**	1.3061*e + *03
	Min	**1.3000*e + *03**	1.3004*e + *03
	Mean	**1.3001*e + *03**	1.3006*e + *03
	Var	**7.4041*e*** − **04**	2.9913*e* − 01

*f*_14_	Max	**1.4001*e + *03**	1.4493*e + *03
	Min	**1.4000*e + *03**	1.4005*e + *03
	Mean	**1.4000*e + *03**	1.4009*e + *03
	Var	**2.7722*e*** − **04**	2.8527*e + *00

*f*_15_	Max	**1.5015*e + *03**	1.9050*e + *05
	Min	**1.5004*e + *03**	1.5026*e + *03
	Mean	**1.5008*e + *03**	1.5816*e + *03
	Var	**0.0731**	2.7233*e + *03

*f*_16_	Max	**1.6026*e + *03**	1.6046*e + *03
	Min	**1.6001*e + *03**	1.6019*e + *03
	Mean	**1.6014*e + *03**	1.6024*e + *03
	Var	**0.3295**	3.6883***e*** − 01

*f*_17_	Max	**3.4698*e + *03**	8.4770*e + *06
	Min	**1.7150*e + *03**	2.0097*e + *03
	Mean	**2.2377*e + *03**	2.1095*e + *04
	Var	**1.9496*e + *05**	2.0329*e + *05

*f*_18_	Max	**1.1217*e + *04**	6.6050*e + *08
	Min	**1.8094*e + *03**	1.8288*e + *03
	Mean	**3.2529*e + *03**	1.9475*e + *05
	Var	**5.4030*e + *06**	1.0139*e + *07

*f*_19_	Max	**1.9025*e + *03**	1.9555*e + *03
	Min	**1.9000*e + *03**	1.9028*e + *03
	Mean	**1.9011*e + *03**	1.9036*e + *03
	Var	**0.6471**	1.4209*e + *00

*f*_20_	Max	**2.0095*e + *03**	1.2708*e + *08
	Min	**2.0003*e + *03**	2.0241*e + *03
	Mean	**2.0025*e + *03**	4.5834*e + *04
	Var	**3.7953**	2.1988*e + *06

*f*_21_	Max	**2.2435*e + *03**	2.6897*e + *07
	Min	**2.1000*e + *03**	2.2314*e + *03
	Mean	**2.1591*e + *03**	7.4587*e + *03
	Var	**3.7630*e + *03**	2.8735*e + *05

*f*_22_	Max	**2.2207*e + *03**	3.2211*e + *03
	Min	**2.2000*e + *03**	2.2314*e + *03
	Mean	**2.2064*e + *03**	2.2687*e + *03
	Var	85.7389	**5.1234*e + *01**

*f*_23_	Max	**2.6295*e + *03**	2.9923*e + *03
	Min	**2500**	**2.5000*e + *03**
	Mean	2.6208*e + *03	**2.5015*e + *03**
	Var	1.0788*e + *03	**1.7156*e + *01**

*f*_24_	Max	**2.5213*e + *03**	2.6369*e + *03
	Min	**2.5088*e + *03**	2.5251*e + *03
	Mean	**2.5149*e + *03**	2.5338*e + *03
	Var	12.8783	**1.1715*e + *01**

*f*_25_	Max	**2.7015*e + *03**	2.7327*e + *03
	Min	**2.6000*e + *03**	2.6635*e + *03
	Mean	**2.6657*e + *03**	2.6894*e + *03
	Var	1.2703*e + *03	**1.2571*e + *01**

*f*_26_	Max	**2.7002*e + *03**	2.7116*e + *03
	Min	**2.7000*e + *03**	2.7002*e + *03
	Mean	**2.7001*e + *03**	2.7003*e + *03
	Var	**9.1541*e*** − **04**	3.5003***e*** − 01

*f*_27_	Max	**3.1009*e + *03**	3.4144*e + *03
	Min	**2.7004*e + *03**	2.7054*e + *03
	Mean	2.8927*e + *03	**2.7219*e + *03**
	Var	1.9303*e + *04	**6.1325*e + *01**

*f*_28_	Max	**3.2796*e + *03**	4.8154*e + *03
	Min	3.1597*e + *03	**3.0000*e + *03**
	Mean	3.1994*e + *03	**3.0065*e + *03**
	Var	1.2209*e + *03	**5.3483*e + *01**

*f*_29_	Max	**6.6281*e + *03**	6.4392*e + *07
	Min	**3.1309*e + *03**	3.3287*e + *03
	Mean	**3.4966*e + *03**	2.8663*e + *04
	Var	**5.1852*e + *05**	8.6740*e + *05

*f*_30_	Max	**4.2010*e + *03**	1.1393*e + *06
	Min	**3.4416*e + *03**	3.6416*e + *03
	Mean	**3.5937*e + *03**	4.1746*e + *03
	Var	2.8657*e + *04	**1.8202*e + *04**

**Table 8:** The comparison results of optimal solutions for the welded beam design.

Algorithms	*x*_1_	*x*_2_	*x*_3_	*x*_4_	*f*(*x*)
ICSO	**0.205730**	**3.470474**	**9.036624**	**0.2057296**	**1.724852**
HFPSO [4]	—	—	—	—	**1.724852**
EPSO [37]	—	—	—	—	1.724853
MBA [38]	0.205729	3.470493	9.036626	0.205729	1.724853

**Table 9:** The statistical results for the welded beam design.

Algorithms	Worst	Mean	Best	SD
ICSO	**1.724852**	**1.724852**	**1.724852**	6.7089*e − *12
HFPSO [4]	1.974449	1.727370	**1.724852**	2.50*e − *02
EPSO [37]	1.747220	1.728219	1.724853	5.62*e − *03
MBA [38]	1.724853	1.724853	1.724853	**6.94*e − *19**

## Data Availability

All data generated or analyzed during this study are included in this published article. Color versions of one or more of the figures in this paper are available from the corresponding authors upon reasonable request.
